The article "A Real-Time Detection Algorithm of Flame Target Image" was retracted in 2023. Reasons: signs of a paper mill; suspected computer-generated content; unreliable results or conclusions; concerns about the data.

# A Real-Time Detection Algorithm of Flame Target Image

**DOI:** 10.1155/2022/5277805

**Published:** 2022-10-11

**Authors:** Jing Zhao

**Affiliations:** School of Computer Science and Engineering, Nanjing University of Science & Technology, Nanjing 210094, China

## Abstract

In many research tasks, the speed and accuracy of flame detection using supply chain have always been a challenging task for many researchers, especially for flame detection of small objects in supply chain. In view of this, we propose a new real-time target detection algorithm. The first step is to enhance the flame recognition of small objects by strengthening the feature extraction ability of multi-scale fusion. The second step is to introduce the *K*-means clustering method into the prior bounding box of the algorithm to improve the accuracy of the algorithm. The third step is to use the flame characteristics in YOLO+ algorithm to reject the wrong detection results and increase the detection effect of the algorithm. Compared with the YOLO series algorithms, the accuracy of YOLO+ algorithm is 99.5%, the omission rate is 1.3%, and the detection speed is 72 frames/SEC. It has good performance and is suitable for flame detection tasks.

## 1. Introduction

Fire is one of the natural disasters closest to people's daily life, and its influence is well known, which will have an incalculable impact on the safety of people's lives and properties if it occurs [1]. Therefore, there are many various devices for fire prevention, for example, the satellite-based LIDAR can be used in flame temperature detection and the flame color can be used to detect the degree of flame combustion. All these methods have some limitations and have higher requirements for equipment, suitable for the detection of a wide range of areas.

In recent years, with the continuous development of deep convolutional neural networks, their applications have become more and more extensive, including object recognition [2], action recognition [3], pose estimation [4], neural style transfer [5], and flame prevention [6]. Meanwhile, convolutional neural networks have achieved better results in flame detection applications. For example, Chaoxia et al. [7] proposed a single-map flame detection method, which was optimized on Mask R-CNN, enabling better detection results for large flame detection. Jie and Chenyu [8] detected the flame region by optimizing Fast R-CNN, which improved the accuracy of flame detection but had high requirements for flame environment. Wen et al. [9] proposed a new flame detection model, which mainly compared the lightness of the algorithm, and the detection speed rose, but the accuracy was significantly lower. In view of the limitations of the algorithms proposed by many research scholars, i.e., the detection of flame hazards cannot be performed in real time, we propose a new real-time flame hazard detection algorithm model YOLO+. This method solves the untimely flame hazard detection, slow transmission speed, and low detection accuracy. At the same time, the algorithm has a better detection effect of small flame objects with good small object detection capability.

## 2. Related Work

### 2.1. YOLO

YOLO (You Only Look Once) [10, 11] was proposed at the beginning with the advantage of fast speed, and then a series of algorithms have been proposed continuously, and it was subsequently developed into a series of algorithms such as YOLOv2, YOLOv3, and YOLOv4 [12]. It has made a great contribution to the object detection algorithm [13]. In this paper, the XX-net algorithm was optimized on the basis of YOLOv3 to achieve detection of flame object pairs [14]. As shown in Figure 1, the backbone network model structure of YOLOv3, Darknet-53, is shown, with 8, 16, and 32-fold downsampling, respectively, so as to perform information splicing and feature information fusion. Also, three different kinds of multi-scale feature information of 52 × 52, 26 × 26, and 13 × 13 were fused to improve the algorithm's feature extraction capability for different scale information [15]. Although the proposed YOLOv3 has achieved some effect on improving the accuracy of the object detection algorithm, YOLOv3 is less effective for small object detection [16]. Especially, when detecting flames in small areas, YOLOv3 is not effective in preventing flame spread [17]. For this reason, we proposed the flame object detection algorithm XX-net based on the YOLOv3 algorithm [18].

### 2.2. Small Object Flame Region

The backbone of the YOLOv3 algorithm is Darknet-53 [19], which has a small shallow feature grid area during feature extraction and provides output for location information, most notably 13 × 13, 26 × 26, and 52 × 52 fusion methods, resulting in a minimum resolution scale feature of 52 × 52 size.

However, the output of the algorithm is 416 × 416 images, so the network division is not refined enough, and some information will be lost in the process of continuous iterative calculation, resulting in a more obvious phenomenon of information loss in some feature maps.

There is some missing information in the flame object detection, resulting in inaccurate flame detection for small objects. The deep grid information region is divided into larger areas, which provides greater semantic information, so it is more effective for large object flame detection, as shown in Figure 1.

In order to improve the feature extraction capability of the YOLOv3 small object detection algorithm and the ability to identify small object flame recognition better and faster, we added the scale grid with smaller resolution to fully extract the information of the feature map [20]. However, with the increase of extracted feature map small object information, the computational and parametric quantities of the algorithm model also increase and the running speed of the network model decreases. Therefore, in this paper, a grid with a model scale of 104 × 104 is added for feature extraction of small objects.  Figure 2 shows the structure of the improved YOLOv3 network model.

In the first step, we calculated convolution and upsampling for layer 74 (L74). The size of the 1st scale feature map was 13 × 13, and the feature fusion operation was performed on the 26 × 26 sized feature map of the layer 61 in the output 13 × 13 sized feature map. The 26 × 26 sized feature map is named as the 2nd scale feature.

In the second step, we fused the 26 × 26 sized feature map of the 2nd scale with the layer 36 output value to obtain the 3rd scale result with the feature map size of 52 × 52.

In the third step, we fused the 52 × 52 sized feature map of the 3rd scale with the layer 11 output value to get the 4th scale result with the feature map size of 104 × 104.

Through the above three steps, we got the new flame object detection algorithm and improved the small object flame detection at the same time.

### 2.3. YOLOv3 Validation Frame Setup

YOLOv3 also sets the prior bounding box to a more meshed model [18, 21–24]. When the flame object is in the grid we set, then this grid is responsible for predicting the class of this object value while labeling it. The prior bounding box of the flame object is shown in Figure 3. The black dotted part of the figure is the central part of the flame. The prior bounding box where the dot is located is responsible for detecting and identifying the flame.

It can be seen from Figure 3 that the size of the prior bounding box in the flame detection area is constant, but the actual size of the detected flame is changeable. Therefore, we further optimized the flame prior bounding box to make the size of the prior bounding box closer to the real flame object. We proposed to use *K*-means algorithm to count the actual prior bounding box size of flame dataset, the number of *K* prior bounding boxes, and the ratio between the length, width, and height of the flame of clustering and the actual flame size [25–27]. *K*-means Euclidean distance was used to calculate the distance of the prior bounding box. As is known to all, the error and the large prior bounding box increase, and the error generated by the algorithm is proportional to the size of the flame prior bounding box. Therefore, we made the intersection ratio of the prior bounding box and the flame actual object detection prior bounding box greater. As shown in formula (1), we used *I* as the distance value.

(1) $$\begin{array}{c} d\left(b,c\right)=1-I\left(b,c\right)\text{,} \end{array}$$

where *b* is the value of any prior bounding box and *C* is the midpoint of the flame prior bounding box. *K*-means algorithm was used to calculate the correlation between *I* and *K*, as shown in Figure 4.

It can be seen from Figure 4 that the horizontal and vertical coordinates, respectively, represent the *K* and *I* values of prior bounding box of flame [28–32]. With the continuous increase of *K* value, *I* value also keeps increasing. We set the number of prior bounding boxes *K* to 12, so 12 clustering center values will also be generated, and the obtained values are shown in Table 1. The obtained clustering center coordinate is proportional to the image size, and the value of the prior bounding boxes can be obtained by convolution operation with the image size of 416 × 416 pixels. Finally, we arrange customers according to the size to form the value in Table 1.

Our improved algorithm is designed with four kinds of feature map information, and we match the feature map of each size scale with three values of prior bounding boxes. For example, the receptive field of the feature map with the size of 13 × 13 was the largest, so it was suitable for detecting the flame region of a large area. We matched it with 208 × 312, 179 × 175, and 121 × 295 prior bounding boxes of a large scale. At the same time, the information of the 26 × 26 feature map was matched with the values of the prior bounding boxes of 117 × 95, 104 × 145, and 71 × 211 sizes. For the same reason, information of 52 × 52 feature map uses values of prior bounding boxes of 62 × 95, 58 × 53, and 46 × 150 in size. The 104 × 104 feature map we added had the smallest receptive field value, which enhanced the detection effect of the algorithm on small-scale flame area. Therefore, we matched the values of 29 × 78, 29 × 36, and 17 × 24 prior bounding boxes for the 104 × 104 feature map.

### 2.4. Feature Extraction

It is known from experience that the scintillation rate of flame is about 8 Hz [33–36]. Therefore, we used the continuous pixel value changes of each frame in the video to extract the flicker characteristic information of the flame center. This method can effectively solve the problem of missed detection rate and misjudgment rate in flame feature recognition. We used the accumulative difference method of luminance value between adjacent video frames to calculate the flame flicker rating, and we established the flicker matrix *M* (*x*, *y*, *t*) and flame luminance value matrix *I* (*x*, *y*, *t*). The calculation formula is shown in formula (2), where *I* (*x*, *y*, *t*) is the brightness value of the flame area of the flame pixel point (*x*, *y*) at *t*; *M* (*x*, *y*, *t*) is the flame video scintillometer value when the flame pixel point (*x*, *y*) is at *t*; and *T* represents the threshold of flame brightness difference between two adjacent frames. When the flame flickers, Δ*I* exceeds the threshold *T*, and the corresponding flame flicker count is increased by 1; otherwise, it remains unchanged.

(2) $$\begin{array}{c} \left\{\begin{array}{c} M\left(x,y,t\right)=\left\{\begin{array}{c} M\left(x,y,t-1\right)+1,∆I>T\text{,}\\ M\left(x,y,t-1\right),other\text{,} \end{array}\right.\\ ∆I=\left|I\left(x,y,t\right)-I\left(x,y,t-1\right)\right|\text{.} \end{array}\right. \end{array}$$

As shown in formula (3), we judge whether it conforms to the characteristic information of flame flicker through the flicker rating rate and times of pixel point *t* for a period of time at time *T*. We usually set the frame *T* of flame flicker as 1 s. If the flame flicker rating rate or time exceeds the threshold *T*_*M*_, the flame in this area is considered to flicker. Finally, we calculate the flicker frequency and number of flame image (*F*) for a period of time, as shown in formula (4).

(3) $$\begin{array}{c} M\left(x,y,t\right)-M\left(x,y,t-T\right)>T_{M}\text{,} \end{array}$$

(4) $$\begin{array}{c} F=\frac{M\left(x,y,t_{n}\right)-M\left(x,y,t_{1}\right)}{t_{n}-t_{1}}\text{.} \end{array}$$

### 2.5. Real-Time Flame Detection

We designed the algorithm flowchart, as shown in Figure 5, designed the flame detection method through six steps, trained the flame detection network by establishing the dataset, and then detected the flame video image by verifying the accuracy of the flame algorithm. The flame detection object was obtained, and the speed and accuracy of video flame detection were analyzed. Finally, the characteristics of flame flicker were used for re-detection and verification.

We used the improved YOLO+ algorithm to output features of segmented images and used the four-scale feature image fusion method as shown in Figure 6 to realize real-time flame image detection. Finally, we used the flicker characteristics of flame to reduce the rate of missing flame detection, thus improving the flame detection effect.

## 3. Experimental Process

### 3.1. Experimental Settings

The experiment was carried out using Ubuntu 20.04 system with a graphics card of 3090 24G and PyTorch 1.6.0 GPU version as the deep learning framework. The size of each image input network model was set to 416 × 416, the number of images input each time was set to 64, and the initial learning rate was set to 0.001.

### 3.2. Dataset

The dataset details we used are shown in Table 2.

We have 6,090 training datasets, 1,060 verification datasets, and 23,354 test datasets, accounting for 30,504 datasets in total, as shown in Figure 7. Our training datasets include flame images and non-flame images, respectively.

### 3.3. Flame Recognition Experiment of YOLO+ Algorithm

In order to verify the effectiveness of network model YOLO+, we conducted experiments on YOLO+, and the test results are shown in Figure 8.

In order to further verify the effectiveness of network model YOLO+, precision rate *A*, false detection rate *P*_*f*_, and missed detection rate *N*_*f*_ are used as evaluation indexes of the algorithm. The calculation method is shown in the following formula:

(5) $$\begin{array}{c} \left\{\begin{array}{c} A=\frac{T_{P}+T_{N}}{N_{pos}+T_{neg}}\times 100\%\text{,}\\ P_{f}=\frac{F_{P}}{N_{neg}}\times 100\%\text{,}\\ N_{f}=\frac{F_{N}}{N_{pos}}\times 100\%\text{,} \end{array}\right. \end{array}$$

where *N*_pos_ represents the number of flame images, *N*_neg_ represents the number of non-flame images, TP represents the number of flame images correctly recognized, TN represents the number of non-flame images correctly recognized, FP represents the number of incorrectly detected flame images, and FN represents the number of missed flame images.

Using the algorithm YOLO+, the accuracy of flame is 99.1%, the false detection rate is 2.5%, and the missed detection rate is 0.8%. Therefore, the algorithm is suitable for fire detection tasks.

The flame detection algorithm designed in this paper has the detection effect as shown in Figure 9, and the marks in the figure represent the detection effect. It can be seen from the experiment that the main reason for the false detection is the interference of external factors on the flame, such as light and sunlight. Therefore, we introduce the flame flicker feature, so as to exclude non-flame images, increase the accuracy of flame detection, and reduce the rate of flame detection. The detection data are shown in Table 3. The accuracy rate is 99.1%, the false detection rate is 2.5%, and the missed detection rate is 0.8%, achieving a good flame detection effect.

### 3.4. YOLO+ Flame Detection Effect

The characteristics of flame flicker were studied in this paper, and Cases 5, 7, 9, and 10 were tested by calculating the frequency of each flame detection effect. The time frequency of flame detection was extracted at an interval of 10 s, and the experimental results are shown in Figure 10. It can be seen from Table 3 that the flicker frequency of Case 5 fluctuates around 8, and the normal flame flicker frequency is around 8, which can be considered as flame. In Case 7, 5 s or so can be considered as a flame image. When the frequency is lower than 7 Hz, we consider the image as a non-flame image. In Case 9, the maximum flame flicker frequency is less than 7 Hz, so Case 9 is regarded as a non-flame image. Similarly, the flicker frequency in Case 10 is between 5 and 9 Hz, so the flame image is excluded.

By using the method in this paper, we effectively reduced some non-flame interference to the flame image. The flame detection effect of algorithm YOLO+ is shown in Table 4.

### 3.5. Comparison of Experimental Results

In order to further verify the flame detection effect of YOLO+ algorithm, experimental comparisons were made between YOLO+ and Faster R-CNN, YOLO, YOLOv2, YOLOv3, YOLOv4, and FCOS. It can be seen from Table 5 that the accuracy of algorithm YOLO+ reaches 99.5%, which is the best, 16.9% higher than Faster R-CNN and 2.5% higher than FCOS. The false detection rate of algorithm YOLO+ is only 1.3%, which is 10 to 20 times lower than that of other algorithms. Therefore, this algorithm greatly reduces the false detection effect of flame images. In addition, our algorithm still performs better than other network models in flame detection speed, which is the same as YOLOv3, but our precision and false detection rate are far lower than those of YOLOv3. Therefore, we finally conclude that YOLOv+ is suitable for flame object detection.

## 4. Conclusion

The frequent occurrence of fire requires higher and higher flame detection, especially for small-scale flame objects. In view of this, we propose a new flame object detection algorithm YOLO+ through YOLOv3 algorithm. Multi-scale detection, *K*-means algorithm, and elimination of some missed flame detection objects are introduced, respectively, to improve the accuracy and speed of the algorithm. Compared with YOLO series of flame detection algorithms, the accuracy of YOLO+ flame detection is 99.5%, the missed detection rate is 1.3%, and the detection speed is 62 frames/s. The algorithm has good performance and is suitable for flame object detection.

## Figures and Tables

**Figure 1:** Structure diagram of YOLOv3 network model.

**Figure 2:** Structure diagram of YOLOv+ network model.

**Figure 3:** YOLOv3 flame verification block diagram.

**Figure 4:** Curve of flame image *K* and *I*.

**Figure 5:** Flame detection process of video image.

**Figure 6:** YOLO+ flame feature map.

**Figure 7:** Partial flame dataset. (a) Dataset of flame images. (b) Dataset of non-flame images.

**Figure 8:** YOLO+ algorithm test effect diagram.

**Figure 9:** Improved YOLO+ flame detection effect diagram.

**Figure 10:** Flame flicker frequency curve.

**Table 1:** Comparison of flame center coordinates and size of prior bounding boxes.

Flame center	Center coordinates	Prior bounding box	Pixel size
0	(0.14, 0.24)	0	17 × 26
1	(0.03, 0.04)	1	29 × 36
2	(0.06, 0.18)	2	29 × 78
3	(0.28, 0.70)	3	46 × 150
4	(0.10, 0.35)	4	58 × 53
5	(0.24, 0.35)	5	62 × 95
6	(0.16, 0.50)	6	71 × 211
7	(0.27, 0.22)	7	104 × 145
8	(0.42, 0.41)	8	117 × 95
9	(0.06, 0.09)	9	121 × 294
10	(0.13, 0.12)	10	179 × 174

**Table 2:** Dataset details.

Dataset	Positive sample image	Negative sample image	Total
Training set	4470	1620	6090
Validation set	650	410	1060
Testing set	15842	7512	23354
Total	20962	9542	30504

**Table 3:** Detection results of flame video and non-flame video.

Flame results						Non-flame results				
Case no.	Total frames	Correct detection	Precision rate (%)	Missed detection	Missed detection rate (%)	Case no.	Precision rate (%)	False detection rate (%)	Precision rate (%)	Precision rate (%)
1	641	643	97.9	6	1.1	7	2885	2.4	98.8	99.4
2	1401	2075	94.4	23	1.6	8	1925	0.0	98.5	97.3
3	1209	2079	94.4	20	1.9	9	540	6.1	98.6	99.3
4	6865	4923	96.1	51	0.9	10	698	16.4	99.4	98.2
5	3194	2957	97.8	37	1.2				98.4	99.7
6	1246	1929	98.2	17	0.8				98.1	98.2

**Table 4:** Flame test data.

Case no.	Total frames	Falsely detected frames	False detection rate (%)
7	3975	0	0
8	3225	0	0
9	650	4	0
10	768	95	8.31

**Table 5:** Comparison of algorithm data.

Algorithm	Precisionrate (%)	False detectionrate (%)	Detectionspeed (frame)
Faster R-CNN	82.6	20.8	39
SSD	89.7	20.7	37
YOLO	93.7	17.2	53
YOLOv2	95.4	15.4	65
YOLOv3	96.2	14.3	72
YOLOv4	96.4	14.1	65
FCOS	97.0	10.0	70
YOLO+	99.5	1.3	72

## Data Availability

The datasets used and/or analyzed during the current study are available from the corresponding author on reasonable request.
